The article "Modulator effect of mangiferin on biochemical characterization in 7,12‐dimethylbenz[a]anthracene induced oral cancer in experimental hamsters" was retracted in 2024. Reasons: unreliable results or conclusions; concerns about the peer review.

# Modulator effect of mangiferin on biochemical characterization in 7,12‐dimethylbenz[a]anthracene induced oral cancer in experimental hamsters

**DOI:** 10.1002/vms3.500

**Published:** 2021-05-05

**Authors:** Min Liu, Chengquan Wen, Shengqi Pan

**Affiliations:** ^1^ Department of Pharmacy Qingdao Municipal Hospital Qingdao China; ^2^ Department of Intensive Care Medicine Qingdao Municipal Hospital Qingdao China

**Keywords:** antioxidant, chemo‐preventive, detoxifying agent, DMBA, lipid peroxidation, mangiferin, oral cancer

## Abstract

**Background:**

Newly, chemo‐preventive technique might be a hopeful advancement in developing countries for treating cancers with the aid of toxic less natural based constituents. Malignancy urges to augment effectual chemo‐preventive agents that are look forward to suppress the tumours which may be stimulated by chewing and smoking of tobacco and over alcohol consumption related with the high prevalence of human oral cancer (OC) patients.

**Methods:**

In the present research, we examined to assess antioxidants, lipid peroxidation (LPO) and detoxification enzymes levels of anticancer activity of mangiferin on 0.5% 7.12‐dimethylbenz[a]anthracene (DMBA) provoked hamster cheek pouch carcinoma (HCPC). OC on hamster buccal pouch (HBP) was incited by DMBA treatment for thrice per week for over 14 weeks.

**Results:**

100% well defined OC establishment with body weight (bw), tumour burden (TB), antioxidant, LPO and liver marker enzymes and also histological changes were observed on DMBA‐challenged buccal pouch carcinoma (BPC) in hamsters. Orally treated mangiferin at an effective dosage of 50 mg/kg bw, to DMBA painted hamsters were significantly averted the body weight, succession of tumour, the biochemical as well as histopathological changes.

**Conclusion:**

Findings of this work clearly suggest that the anti‐carcinoma effect of mangiferin possesses the modulator effects on potent antioxidant, anti‐LPO and detoxification agents to expel the metabolites of malignant cells, on DMBA‐provoked BPC in hamsters.

## Graphical abstract

Orally treated mangiferin at an effective dosage of 50 mg/kg bw, to DMBA painted hamsters were significantly averted the body weight, succession of tumor, the biochemical as well as histopathological changes. Anti‐carcinoma effect of mangiferin possess the modulator effects on potent antioxidant, anti‐LPO and detoxification agents to expel the metabolites of malignant cells, on DMBA‐provoked BPC in hamsters.

## 1 INTRODUCTION

Mouth cancer, a class of head and neck carcinoma (HNC), is a major one and most common malignant condition on global population (Kulasinghe et al., 2018). Oral squamous cell carcinoma (OSCC), by means of changeover from an epithelial to a mesenchymal phenotype, are hallmark in the competence of self‐regulating tumour cell growth towards migrate, invade and metastasize (Clark & Vignjevic, 2015). Therefore, 80% of patients has suffered from oral cancer through widespread exposures for the stimulation and progression of mouth carcinoma like excess alcohol consumption, tobacco smoking and chewing. Although widespread development over finding and progression on behaviour approach, OSCC at rest together drastically augmented death rate and morbidity as well (Niaz et al., 2017). Furthermore, to primary anticipation via the removal of tobacco expenditure, chemoprevention of OC has gained momentum in current years.

Chemo‐prevention practice might be an endowed improvement in developing countries of the world for the treatment of carcinogenesis. A chemo‐prevention, an emerging technique, was covenant with the suppression of malignant growth with the aid of natural herbal‐based compounds (Steward & Brown, 2013). The carcinogenesis suppression capacity of herbal founded phytoconstituents is necessitated to explore by adopting the well established in vivo system as well as evidence suggests that the majority used animal models in oral cancer investigate are the male golden Syrian hamster cheek pouch (HCP) with DMBA (Sun et al., 2008; Warner et al., 2014). DMBA is polycyclic aromatic hydrocarbons contains large class of compounds presenting powerful carcinogen, cocarcinogen and tumour promoters. The cause of these carbon molecules is usually noticeable via degradation/loss of nuclear contents, which when nor repaired and in stagnant mutations of trouble genes originating their multiplication (Bolognesi et al., 1991). Hence, in our research we adopted a DMBA provoked mouth cancer model on hamsters which involves a typical administration of DMBA in thrice per week for over 14‐week regimen. OC induced by DMBA in the HCP protocols in this model induce premalignant changes and carcinomas reiterate many of features that look a lot like human OSCC, which give out as an outstanding target organ for chemo‐intervention for the purpose that of easy convenience and follow‐up of lesions Shklar (1999).

Mangiferin is a natural polyphenol derived from edible herbals, and it was distributed on numerous components of *Mangifera indica* as well as the fruit peelings, stalk, leaf, bark and kernel of mango tree. Mangiferin demonstrated various cellular and experimental models experimentally evaluated its effective function on different malignancies and other ailments (Matkowski et al., 2013). Mangiferin acquired an assured pharmacological activity like antioxidant, anticancer, antidiabetic, antioxidative, immunomodulatory and hepatoprotective effects in various diseases (Du et al., 2018). There is good proof for the chemo‐preventive activity of mangiferin in rodent models, in which it have been shown to inhibit tumour growth in mouse metastatic melanoma, (Takeda et al., 2016) hepatic tumour growth in murine, (Tan et al., 2018) lung carcinogenesis in Swiss albino mice, (Rajendran, Ekambaram & Sakthisekaran, 2008) lung injury in mice, (Wang et al., 2015) dermatitis in a mice (Zhao et al., 2017). It also suppressed human breast cancer cells (Louisa et al., 2014). In our research work, we planned to explore the relative antioxidant capacity of mangiferin (50 mg/kg bw), an effective dose for inhibitory efficacy on DMBA‐challenged HBPC. The different parameters were adopted to investigate the chemo‐preventive efficacy of mangiferin against DMBA‐provoked mouth cancer in hamster model.

## 2 MATERIALS AND METHODS

### 2.1 Chemicals and reagents

Mangiferin (Figure 1a) DMBA and liquid paraffin (LP) were purchased by sigma Aldrich chemicals Pvt. Ltd (US). The entire erstwhile chemicals were adopted of diagnostic status, obtained from Hi‐Media Lab Pvt. Ltd. (US).

**FIGURE 1:** (a) Structure of mangiferin and (b) experimental protocol for effective dose study

### 2.2 Animals

Eight‐ to 10‐week aged hamsters (*Mesocricetus auratus*), weighing about 80–120 g, were maintained in the central animal house. They were residence five propylene cages; all cage limited 6 hamsters were maintained separately and had access to pelleted diet with H_2_O ad libitum. Hamsters were housed in guarded situation with 27°C ± 2°C temperature and 55% ± 5% moistens with a 12‐hr light/dark series.

### 2.3 Experimental design

Whole set of animals (24 hamsters) were alienated into 4 groups with six hamsters in each. Figure 1b shows in the experimental design for effective dose study. Group I hamsters were supplied as normal control animals. Groups II and III hamsters were treated with 0.5% DMBA in LP three times for a week to 14‐week regimen in their gone HBP using a number four brush. Group III hamsters received in orally pretreatment with 50 mg/kg body weight of mangiferin, suspended on corn oil, starting 1 week prior to the disclosure of carcinogen and sustained in alternate periods to DMBA challenge in the end of 14 weeks. Oral treatment of 50 mg/kg bw/day of mangiferin was given to Group IV hamsters in unaccompanied during the study regimen. The experimentations were finished on 10th week, and every hamster was killed after anaesthetization via displacement of cervical bone.

Body weight of studied hamsters was measured by means of subtraction of earlier and final body weight. Collected hamster's plasma was utilized for biochemical studies and liver and cheek pouch tissues were exploited for Histopathological examine, for this collected cheek pouch was immediately trenched on formalin solution and the processed tissues were implanted in paraffin wax, pieces were sliced with the aid of microtome and coloured by haematoxylin and eosin (H&E) were conducted on untreated control and treated hamsters.

### 2.4 Tumour assessment

Total tumours on every HCP were inspected macroscopically, then hamsters were euthanized and width of every tumour was calculated with the aid of vernier metre. The volumes of tumours were determined by applying the formula of *V* = 4/3π (D1/2) (D2/2) (D3/2) where D1, D2 and D3 means the three widths (mm3) of tumour. The TB was proposed via multiplication of the volume of tumour and tumour numbers for each HBP.

### 2.5 Biochemical analysis

#### 2.5.1 Sample collection

After anaesthetic hamsters killed, the blood was gathered on heparin painted containers and utilized to separate the plasma by spinning the tube at 18 *g* for 20 min. Liver and HBP tissues were detached and cleaned by icy buffered saline pulverized to become homogenize and then the homogenized suspensions were utilized for biochemical investigations.

Total protein substances were calculated approximately by adopting the Lowry et al. method (Lowry et al., 1951). For confirming the generation of TBARS, LOOH and CD on plasma and oral mucosa, the lipid peroxidation was determined by applying the method of Ohkawa et al. (1979), Jiang et al. (1992) and Rao and Recknagel (1968) in that order. Enzymatic functions of SOD, GPx, CAT content on the plasma and buccal mucosa were calculated by the procedure of Kakkar et al. (1984), Rotruck et al. (1973) and Sinha (1972) in that order. GSH and Vit‐E levels on plasma and buccal mucosa were resolute with the procedure of Beutler and Kelly (1963), Desai (1984) and Palan et al. (1991) correspondingly.

Liver marker enzymes like cyt‐p450 and cyt‐b5, DTD, GST, GR, GSH and GSSG levels on liver and oral mucosal tissues were established by adopting the procedure of Omura and Sato (1964), Lind et al. (1990), Habig et al. (1974), Carlberg and Mannervik (1985), Anderson (1985), Tietze (1969) and Ernster et al. (1967) accordingly. Protein detection was done with the aid of Bradford protein detection colorimetric kits (Bio‐Rad, CA).

#### 2.5.2 Statistical analysis

The data was illustrated as mean ± *SD*. Biochemical parameters were executed with one‐way ANOVA afterwards DMRT for the comparison by statistically. The results were judged statistically significant if *p* < 0.05.

## 3 RESULTS

### 3.1 Effect of mangiferin on body weight of hamsters

The body weight was précised as changes involving, starting and finishing period of control and treated hamsters were depicted. Significant (*p* < 0.05) depletion on body weight was noted in DMBA induced OSCC, while supplement with 50 mg/kg bw of mangiferin by orally in thrice times for each week for up to 14 weeks exhibited a significant (*p* < 0.05) improvement in body weight gain of DMBA challenged hamsters. Orally preadministration of mangiferin alone hamsters revealed a similar body weight when matched with untreated normal group.

### 3.2 Incidence of oral tumour

Incidences, volume and TB of tumours of normal and studied hamsters were depicted. In our work, hundred percentage tumour development noted by way of mean tumour volume (189.37 mm^3^) and TB (1,704.33 mm^3^) in DMBA induce HBPC. Mangiferin with DMBA treated hamsters significantly (*p* < 0.05) undeveloped the incidence, volume and burden of tumours. Untreated normal hamsters possessed no tumour formation as well as mangiferin alone hamsters.

### 3.3 Histopathological evaluation oral mucosa tissue

The pathological changes observations of oral mucosa of normal and studied hamsters were illustrated in Figure 2. In our work, 100% development of tumour and harsh hyperkeratosis, hyperplasia, dysplasia and well documented OSCC were observed in the cheek pouch epithelium of tumour growth HBP. While well differentiated SCC was not observed on buccal pouch epithelium of DMBA treatment with mangiferin administered hamsters were moderate mild keratosis and hyperplastic epithelium. Oral administration of mangiferin alone and untreated control exhibited clear epithelial deposits.

**FIGURE 2:** (a) Histopathological changes in the oral mucosa of control and experimental hamsters. (b) Photomicrograph showing well differentiated OSCC exhibiting enlarged cells in group 2 DMBA alone hamsters (arrow indicated). (c) Oral mucosa epithelium from group 3 (DMBA + Mangiferin) hamsters showed normal cellular structural design by mild to moderated hyperkeratosis and hyperplasia. (a,d) Group 4 (mangiferin‐alone) and group 1 (control) hamsters showed normal squamous epithelium through no signs of cellular growth

### 3.4 Status of plasma and oral mucosa lipid peroxidation

In Figure 3, explains the level of LPO derivatives of TBARS, CD and LOOH on plasma and cheek pouch of normal and treated hamsters. This work revealed the significant augmentation in lipid peroxidation on plasma and suppressed in the buccal tissues of DMBA challenged hamsters when checked with normal animals. Supplementation of mangiferin by orally to DMBA‐challenged hamsters exhibits near normal level of prominence LPO derivatives in plasma and cheek pouch when checked with normal group, whereas control and mangiferin alone supplemented hamsters possessed no differences.

**FIGURE 3:** The status of lipid peroxidation by‐products in the plasma and buccal mucosa of control and experimental hamsters. Results are expressed as mean ± *SD* for six hamsters in each group. Data not sharing a common superscript letter (a–c) differ significantly at *p* < 0.05 (DMRT)

### 3.5 Enzymatic antioxidant levels of plasma and oral mucosa

Figure 4 demonstrates the levels of enzymatic antioxidant on plasma and oral mucosal tissue of normal and studied hamsters. Enzymatic antioxidant status on plasma and cheek pouch was demonstrated the significant decreased, except for GPx (enlarged) in the oral pouch of hamsters OC. Oral administered with mangiferin to DMBA‐challenged hamsters confirmed the significant (*p* < 0.05) brought back to near normal level of antioxidant enzymes as compared to untreated control, however mangiferin supplemented hamsters demonstrate nil significant variation on enzymatic antioxidant activity as compared with untreated normal group.

**FIGURE 4:** The levels of enzymatic antioxidant in the plasma and buccal mucosa of control and experimental hamsters. Results are expressed as mean ± *SD* for six hamsters in each group. Data not sharing a common superscript (a–c) differ significantly at *p* < 0.05 (DMRT)

### 3.6 Levels of plasma and cheek pouch nonenzymatic antioxidant

Figure 5 illustrates the nonenzymatic antioxidants level of plasma and cheek pouch of untreated normal and treated hamsters. Considerable decrease of nonenzymatic antioxidants of plasma was noted, while they augmented in the cheek pouch of hamsters during OSCC. Preadministered with mangiferin to DMBA‐challenged hamsters revealed significant near normal levels of nonenzymatic antioxidants to both plasma and buccal mucosa when checked with untreated normal group, additionally hamsters treated with mangiferin alone and untreated control possessed none modifications in nonenzymatic antioxidants function.

**FIGURE 5:** The status of nonenzymatic antioxidants in the plasma and buccal mucosa of control and experimental hamsters. Results are expressed as mean ± *SD* for 10 hamsters in each group. Data not sharing a common superscript (a–c) differ significantly at *p* < 0.05

### 3.7 Detoxification marker enzymes level in hepatic tissue

Figure 6 revealed the phase I and phase II hepato‐protective enzymes level in liver tissue of untreated control and treated hamsters. In our study, we detected that the phase I enzyme was enhanced, while phase II enzyme was considerably reduced in HBP tumour formation, but supplementation of mangiferin by orally to DMBA‐challenged treated hamsters remarkably reinstated the phases I and II enzyme. Therefore, mangiferin supplemented hamsters revealed no notable alterations on phases I and II enzyme levels as contrast to untreated control.

**FIGURE 6:** The status of phase I and phase II detoxification enzymesin the liver of experimental hamsters. Results are expressed as mean ± *SD* for six hamsters in each group. Data not sharing a common superscript (a–c) differ significantly at *p* < 0.05 (DMRT)

### 3.8 Oral mucosal level of phases I and II enzymes

Level of phases I and II detoxification enzymes of oral mucosa of untreated normal and treated animals was depicted in Figure 7. Functions of phase I detoxification mediators were remarkably enhanced, whereas phase II altered (GSH/GSSG proportion was elevated; GSSG was suppressed) on HCP carcinogenesis. Supplementation of mangiferin by oral route to DMBA‐challenged hamsters notably regained the enzymatic functions of phases I and II detoxification regulators; though mangiferin in alone supplemented animals possessed nil variations on phases I and II enzymes level.

**FIGURE 7:** The status of phase I and phase II detoxification enzymesin the oral mucosa of experimental hamsters. Results are expressed as mean ± *SD* for six hamsters in each group. Data not sharing a common superscript (a–c) differ significantly at *p* < 0.05 (DMRT)

## 4 DISCUSSION

OC is an major health consequence among the Asian countries and regarded as the widespread neoplasm condition that possessing a huge deleterious effect on well‐being with elevated morbidity and mortality rate (Coelho, 2012). Chemo‐prevention technique was emerged as an preventing and treating of malignancies with the aid of natural‐based herbal constituents (Benetou et al., 2015). In vivo chemo‐preventive and anti‐cancer activities on mangiferin on various cellular and experimental models, it can explore through the inhibition of tumour growth in different treated hamsters models of various cancers. Li et al. (2002) confirmed that the anti‐neoplastic activity inhibition of cell viability and diminishing metastatic stages. DMBA‐induced HBPC was adapted to measuring the chemo‐preventive capabilities of naturally occurring constituents; because DMBA stimulated mouth carcinoma was narrowly exhibiting the mouth carcinoma of humans by histopathologically and as well as morphologically. Our current research, a typical administration of DMBA for 14‐week regimen possessed a well‐built SCC and linked with elevated burden of tumour and also exhibited a harsh hyperplasia, hyperkeratosis and dysplasia. This study revealed the 100% formation of tumour on buccal pouches of DMBA challenged hamsters only, while tumours were histopathologically confirmed with slightly altered squamous cell carcinogenicity.

Tan et al., 2018) reported that mangiferin administrated through orally inhibited orthotopic hepatocellular carcinoma growth in implantation dose dependently suppressed the free expansion in experimental and invasion in vitro model via β‐catenin in Wnt pathway. In our present study, supplementation of 50 mg/kg bw of mangiferin by oral route to DMBA‐challenged hamsters remarkably inhibited and suppressed tumour development. Consequently, our findings signify that mangiferin have significant chemo‐preventive efficiency while DMBA mediated mouth malignancy. Chemo‐preventive prospective of mangiferin may because of its destructive action against neoplasm condition through mouth malignancy.

A chemo‐preventive regulators altered the DNA damaging units to the removable metabolites via excretion by means of instigation of detoxification mediators (Vijayalakshmi and Sindhu (2017), Rajendran, Ekambaram & Sakthisekaran (2008) and Rajendran et al. (2013) postulated that mangiferin (50 mg/kg bw) delayed the tumour developments in mice with no notable alterations of the body mass. Rajendran et al. (2014) and Hu et al. (2013) have found that pretreatment of mangiferin (50 mg/kg bw) for 5 weeks in the Swiss albino mice model in this due explored the suppression tumour growth development. These studies were corroborating with our findings. Shi et al. (2016) has been revealed that mangiferin can kindle up G2/M phase cell cycle detain throughout down regulating Cdc2‐cyclin B1 and induces apoptosis through suppressing human lung cancer cell lines. Further in their studies mangiferin exerts anti neoplastic effects experimental animals, with more potent to drastically diminish the burden and volume of subcutaneously and enlarge A549 xenograft of mice span. An additional work on mangiferin revealed the scavenging efficiency of mangiferin which may benefit to guard the cells beside oxidative stress stimulated injury and mutagenesis. Schwartz and Shklar (1996) established that mediator which stimulate the enzymatic functions of GST possess remarkable chemo‐preventive prospective while formation of cancer. Diminished functions of phase II toxins excreting stimulator was accounted on numerous varieties of cancer development stages in order (DeBerardinis and Chandel (2016). Hence, in our present study, it was confirmed that the orally administered mangiferin with DMBA‐treated hamsters come back the level of phase II toxins removing regulators up to near normal level. This current work disclosed that the mangiferin improved removal and eliminating processes of metabolites of malignant cells while DMBA‐challenged HBPCs.

Generation of ROS and elevated oxidative stress takes a major role in pathological process of different malignancies together with OC. Assessment of TBARS level in serum of plasma was an unfailing indicator to measure injury level of tissues under pathophysiological circumstances. Although, GST and GR were the detoxify DMBA metabolites, further escaped diol epoxide derivatives able to attach with adenine deposits of DNA which causes mutation which endorses the endurance and progression of cells. Magniferin at dose 100 mg/kg bw, medicated mice (C57BL/6J) was confirmed development of tumour than cisplatin, which was explore the mangiferin was good chemo‐preventive mediators (Goldsworthy & Fransson‐Steen, 2002). This study was similar with our findings. TBARS of DMBA‐challenged hamsters revealed the lipid peroxidation depleting potential of mangiferin while mouth malignancy. Peng et al. (2004) reported the suppressive efficacy of mangiferin against blood cancer (k562) cell proliferation, also down regulated the NF‐kB induces programmed cell death. Rajendran et al. (2014) suggested that mangiferin was a potent anticancer agent due to their capability to suppress free radicals.

Improved LPO connected by the way of depleting the antioxidants on passage was key verdict on conversion of malignancy. ROS discharge extremely toxic oxygen molecules, navigate layers and stimulate negative property of this position apart from carcinogenesis (Dreher & Junod, 1996). The better LPO in passage of hamsters challenged with DMBA mouth tumours imitates too much accumulation of free radicals aggravated by diminished competence of defence mechanisms of hosts. The elevation on LPO directly interlinked to the reduction of enzymatic antioxidants. The ascorbic acid (vitamin C) is a major and very important antioxidant which vanishes quicker than any other antioxidants at the time of exposure of plasma to elevated ROS (Frei et al., 1989). Vit‐E is an imperative antioxidant and also a lipid solubilising agent occurs in blood and mucosabuccal tissues (Gerster, 1995). GSH, an important in vitro reluctant, presents defence besides the free radicals, peroxides and other toxic agents (Viña et al., 1989). Insufficiency of vit‐C, vit‐E and GSH in blood of tumour having animals might owing their improved consumption to forage of produces of LPO. The depleted enzymatic functions of GPx, SOD and CAT which are essential toxins removing enzymes of cells was described in carcinogenicity (Fiaschi et al., 2005). These findings was narrowly supported this current work. Supplementation of mangiferin through oral route was regained the alterations which is mediated by DMBA and this finding highlighting the suggestions of chemo‐preventive efficiencies of plant derived constituents.

Mangiferin was mentioned as alter the LPO level while generating the elevated antioxidants. It was already mentioned that the mangiferin can elevate the GSH, GPx, SOD and CAT level (Sellamuthu et al., 2013). This current work exhibited that mangiferin possessed the suppression of tumours through transforming the LPO and antioxidant level on intent organs. Das and Roy (2012) were studied that hepatoprotective effect, which is augmented LPO and lower the levels of cellular GSH in D‐galactosamine (GAL) stimulated hepatotoxicity rats model. Further in his studies showed in the in vitro study liver cells exposed GAL5mM were stimulated the apoptotic condition and cell death with elevated ROS and NO accumulation. Rajendran, Ekambaram, Magesh, et al., (2008)) has been described that oral administrated mangiferin proved excess production of the detoxification regulators, like GSH transferase, quinine reductase and uridine 5’‐diphosphate‐glucoronosyl transferase, hold back the genotoxicity in lung bearing rats.

Findings described above revealed that mangiferin is able to be an effectual chemotherapy drug, and by additional investigations on mangiferin, it can endorse the prevention and treatment of malignancies. ROS have to be removed quickly to evade the cell injuries and necrosis and carcinogenesis as well, this was mediated by the antioxidants via regulation of toxin removing pathway. In this study mangiferin proved as a recognized antioxidant drug that can neutralize and remove the widespread ROS because of the influential expressions, functions as an important toxins removing agents supplied to depletion in oxidative stress. It was previously mentioned that the mangiferin narrowly defends against elevated ROS level mediated by widespread agents (Kawpoomhae et al., 2010). Alongside its free radical scavenging potential, mangiferin power to ROS production by traversing fenton‐type responses.

Fenton‐type responses normally engaged on the hydroxyl radical accumulation and thereby oxidation of Fe 2+ to Fe 3+. With the mangiferin treatment, Fenton‐type responses was refused via connecting the Fe 2+ ions and by restrain the ROS accumulation (Muruganandan et al., 2005). Furthermore, Duang et al. (2011) have done that mangiferin protects against LPO. This defence mechanism might within part accountable for depleted DNA adduct formation and attenuation of cytotoxic functions. Mutually *cellular* and *experimental* confirmations recommend the improved expressions of widespread toxins removing enzymes mediated by mangiferin lead to attenuation of ROS accumulation. In supplement to these findings, (Matkowski et al., 2013) mangiferin prejudiced CAT, SOD and GPx in that order it halt the ROS centred apoptosis via depleting the intercellular accumulation of ROS. Banerjee et al. (2017) revealed the relationship within the mangiferin and GSH through arrangement by mangiferin elevated excessive level of GSH in experimental supplementation with erstwhile antioxidant agents. Sarkar et al. (2004) additionally recommends the efficiency mangiferin to vanish the elevated oxidative stress was may connected with down regulation of NF‐kB, that depletes the TNF‐mediated ROS accumulation. CAT is an essential toxins removing enzyme responsible for antioxidant ability in many organisms possessing oxygen which renovates H_2_O_2_ to H_2_O and O_2_. If H_2_O_2_ was not quickly removed or converted to tiny species, it can stimulate the oxidative injury. Mangiferin was directly escalating the CAT enzyme's efficacy via mutual functions with the enzyme, thereby depleting the oxidative injury that can able to complete in earlier to the removal of H_2_O_2_. The escalated function of CAT could vary downstream pathways which shows that an atmosphere does not endorse carcinogenicity (Ren & Guo, 2018).

Leiro et al. (2003) has demonstrated that mangiferin inhibits the iNOS and TNF‐α gene expression which exhibits mangiferin have therapeutic of inflammatory and hemo‐generative disorder. Yoshimi et al. (2001) showed 50 mg/kg bw, to have in vivo tumour growth suppressive action against AZO enzyme (AOM) induced rats in colon cancer model due to their anti‐cell proliferative activity this property were strongly recommends a mangiferin was potential naturally occurring chemo‐preventive drug. Cuccioloni et al. (2016) postulated that mangiferin has a therapeutic potential to selectivity block breast cancer cell multiplication through striking the multiplication of cells and stimulating apoptosis. These findings were more supported to our present finding suggested on mangiferin have anti‐cancer, anti‐neoplastic and anti‐metastatic properties.

## 5 CONCLUSION

Taken together, the present study thus concludes that protective effect of mangiferin on tumour cell proliferation in DMBA‐induced HBPC. While the mechanism through which mangiferin exerts its prevented DMBA induced OC in the HCP via its anti‐cell proliferative anti LPO and antioxidant possible and also adjusting the prominence of phase I and II hepatoprotective mediators. This study was supportive in determining the dose employed against oral tumours in the development of a new and a potential anticancer drug. It may offer a drug to use in clinical phases needs more investigations on its the molecular means of functions and probable usefulness of Mangiferin as a drug for chemotherapy.

## CONFLICT OF INTEREST

The authors declare no conflict of interest.

## AUTHOR CONTRIBUTION

**Min Liu:** Methodology; Writing‐review & editing. **Chengquan Wen:** Formal analysis; Investigation; Validation.

## ETHICS APPROVAL AND CONSENT TO PARTICIPATE

The study protocols were approved (9982.2019.FLK. Sh/Sh.Q) by the Department of Intensive Care Medicine, Qingdao Municipal Hospital, Qingdao, Shandong, China after critical evaluation.

## HUMAN AND ANIMAL RIGHTS

No human were used for studies that are base of this research. The reported experiments were performed in accordance with the standards set forth in the 8th Edition of Guide for the Care and Use of Laboratory Animals.

## Data Availability

All the data has been presented in this article.
